The article "Study on the Correlation between Chinese Medicine Syndrome and Cognitive Dysfunction in Mild Cognitive Impairment" was published in 2022. Journal: Evid Based Complement Alternat Med.

# Study on the Correlation between Chinese Medicine Syndrome and Cognitive Dysfunction in Mild Cognitive Impairment

**DOI:** 10.1155/2022/7117704

**Published:** 2022-06-24

**Authors:** Zhiying Lin, Tianwen Huang, Guanyi Zheng, Runqiong Chen, Minglong Yao, Wenhong Liu, Shujie Li

**Affiliations:** ^**1**^ Department of Traditional Chinese Medicine, The Affiliated Union Hospital of Fujian Medical University, Fuzhou 350001, China; ^**2**^ Department of Neurology, The Affiliated Union Hospital of Fujian Medical University, Fuzhou 350001, China; ^**3**^ Fujian Mingdong Health School, Ningde 355017, China

## Abstract

**Objective:**

To investigate the correlation between Chinese medicine syndrome and cognitive dysfunction in patients with mild cognitive impairment (MCI).

**Methods:**

121 MCI patients were included for syndrome differentiation and syndrome scoring according to the Chinese medicine syndrome classification standard of senile dementia. The cognitive function and cognitive subitems (including visual space and executive function, naming, attention, language, abstraction, delayed recall, and orientation) of patients with different Chinese medicine syndromes were scored with the Montreal Cognitive Assessment (MoCA). Correlation analysis was made on Chinese medicine syndromes and cognitive domain damage.

**Results:**

Chinese medicine syndromes from most to least were kidney deficiency and marrow reduction syndrome, turbid phlegm obstructing orifices syndrome, deficiency of heart and spleen syndrome, *qi* stagnation and blood stasis syndrome, and *yin* deficiency of heart and liver syndrome. There were no significant differences in MoCA scores among different Chinese medicine syndromes (*P* > 0.05).In the kidney deficiency and marrow reduction syndrome, the delayed recall score was 1.74 ± 1.23 and the difference was statistically significant when compared with deficiency of heart and spleen syndrome or the *yin* deficiency of heart and liver syndrome (*P* < 0.05). In the turbid phlegm obstructing orifices syndrome, the delayed recall score was 1.81 ± 1.33 and the difference was statistically significant when compared with the *yin* deficiency of heart and liver syndrome (*P* < 0.05). There was a significant negative correlation between the kidney deficiency and marrow reduction syndrome's Chinese medicine syndrome scores and MoCA scores (*P* < 0.01), and there was a negative correlation between the turbid phlegm obstructing orifices syndrome's Chinese medicine syndrome scores and MoCA scores (*P* < 0.05). Correlation analysis showed that the kidney deficiency and marrow reduction syndrome was significantly negatively correlated with delayed recall scores (*P* < 0.01), and it was also negatively correlated with visual space and executive function scores (*P* < 0.05). The turbid phlegm obstructing orifices syndrome was significantly negatively correlated with delayed recall scores (*P* < 0.01).

The article "Study on the Correlation between Chinese Medicine Syndrome and Cognitive Dysfunction in Mild Cognitive Impairment" was published in 2022. Journal: Evid Based Complement Alternat Med.

**Conclusion:**

The kidney deficiency and marrow reduction syndrome and the turbid phlegm obstructing orifices syndrome were the most common syndromes in MCI. Patients with kidney deficiency and marrow reduction syndrome might have obvious damage in delayed recall function and have damage in visual space and executive function. Patients with turbid phlegm obstructing orifices syndrome might have obvious damage in delayed recall function.

## 1. Introduction

Mild cognitive impairment (MCI) refers to the transition state between normal and dementia patients, indicating that there is significant memory and/or other cognitive impairment compared to the control group that matches the age and educational level. The daily living ability of MCI is normal, and it does not meet the diagnostic criteria for dementia yet. Studies have shown that MCI prevalence of elderly people over the age of 60 is about 15%–20%, and the conversion rate from MCI to dementia is about 8%–15% annually [1]. MCI includes a variety of reasons, Alzheimer's disease and cerebral small vessel disease are the two main reasons. There is no recognized effective method for the treatment of MCI at present [2]. However, studies have shown that traditional Chinese medicine (TCM) may be effective in the prevention and treatment of MCI [3, 4]. Although there are different opinions on Chinese medicine syndromes of MCI, they mainly focus on kidney deficiency, qi deficiency, blood stasis, and phlegm resistance. This study aims to evaluate the correlation between Chinese medicine syndromes and cognitive dysfunction of MCI and provide an objective basis for Chinese medicine syndrome differentiation and treatment of MCI.

## 2. Subjects and Methods

### 2.1. Diagnostic Criteria for MCI

In accordance with the international MCI working group standards and Chinese guidelines for the diagnosis and treatment of dementia and cognitive impairment, the MCI diagnostic criteria were as follows [5, 6]: first, persons should be judged as not normal besides not fulﬁlling the diagnostic criteria for dementia [7]. Second, functional activities of the persons are mainly preserved, or at least that impairment is minimal. Furthermore, the persons should have evidence of cognitive decline, measured either by a self and/or informant report in conjunction with deﬁcits on objective cognitive tasks, and/or evidence of decline over time on objective neuropsychological tests.

The article "Study on the Correlation between Chinese Medicine Syndrome and Cognitive Dysfunction in Mild Cognitive Impairment" was published in 2022. Journal: Evid Based Complement Alternat Med.

### 2.2. Chinese Medicine Syndrome Differentiation and Classification

Referring to the Chinese medicine clinical research of new drugs guiding principles (2002 edition) [8] for senile dementia clinical research guidelines, five Chinese medicine syndromes were kidney deficiency and marrow reduction syndrome, turbid phlegm obstructing orifices syndrome, *qi* stagnation and blood stasis syndrome, deficiency of heart and spleen syndrome, and *yin* deficiency of heart and liver syndrome. The information of the four diagnoses of the subjects will be analyzed and the Chinese medicine syndromes will be determined by the senior TCM physicians.

### 2.3. Inclusion and Exclusion Criteria

Patients were included if they fulfilled the following criteria: (1) conform to MCI diagnostic criteria and Chinese medicine syndrome differentiation criteria; (2) age ranged from 60 to 80; (3) Clinical Dementia Rating Scale (CDR) scored 0.5; (4) Functional Activities Questionnaire (FAQ) scored < 5 points [9]; (5) provided written informed consent.

Patients were excluded if they had the following: (1) mental and neurodevelopmental retardation; (2) brain tumors, multiple sclerosis, encephalitis, epilepsy, Parkinson's disease, normal intracranial pressure hydrocephalus, and syphilis; (3) liver function insufficiency, renal insufficiency, vitamin deficiency, thyroid dysfunction, etc.; (4) alcohol abuse and drug abuse; (5) Center for Epidemiologic Studies Depression Scale ≥ 16 points [10]; (6) other known diseases to cause cognitive impairment.

### 2.4. Patients

Eligible patients who visited the Department of Traditional Chinese Medicine, Union Hospital Affiliated to Fujian Medical University, from June 2015 to June 2018 were recruited after inquiry of disease history, general physical examination, neurological examination, neuropsychological assessment, and imaging examination (Figure 1). The research plan was approved by the Ethics Committee of Union Hospital Afﬁliated to Fujian Medical University (No. 2013KY020).

### 2.5. Outcome Measures

Neuropsychological tests were performed. All participants underwent the Montreal Cognitive Assessment (MoCA) [11]. MoCA included 8 aspects of visual space and executive functions: naming, memory, attention, language, abstraction, delayed recall, and orientation, with a total score of 30 points. In addition, all participants were assessed by the Functional Activities Questionnaire (FAQ) [9] and the Center for Epidemiologic Studies Depression Scale (CES-DS) (≥16 points were excluded for it suggested depression) [10].

### 2.6. Chinese Medicine Symptom Rating Scale Test

The syndrome differentiation was according to the diagnostic criteria of Chinese medicine syndromes for senile dementia [8]. Patients who have 2 items of main symptoms (necessary for mental retardation), at least 2 items of secondary symptoms, and any 1 item of the tongue and pulse were diagnosed as one certain Chinese medicine syndrome. The symptoms of each syndrome were recorded as 3, 2, 1, and 0 points, respectively, according to the severity, middle, mild, and no symptoms of the disease.

The article "Study on the Correlation between Chinese Medicine Syndrome and Cognitive Dysfunction in Mild Cognitive Impairment" was published in 2022. Journal: Evid Based Complement Alternat Med.

### 2.7. Statistical Analysis

SPSS 18.0 software (Chicago, IL, USA) was used for data analysis. The normality test was carried out in each group and variables of the normal distribution were shown as mean ± standard deviation ($\bar{x}\pm s$). One-way analysis of variance was used to compare the normal distribution of the measurement data, and the LSD-t test was used for comparison between the groups. The Kruskal–Wallis H test was used when measurement data were not normal distribution. Enumeration data were compared by the chi-squared test. Pearson's correlation was used to investigate the correlation between the total scores of each Chinese medicine syndrome and MoCA or its subitems scores. All statistical tests are two-sided probability tests. *P* < 0.05 was considered to be statistically signiﬁcant.

## 3. Results

### 3.1. Comparison of Gender Composition, Age Distribution, and Educational Level of Chinese Medicine Syndromes of MCI

Table 1 shows that the types of Chinese medicine syndromes from most to least were kidney deficiency and marrow reduction syndrome, turbid phlegm obstructing orifices syndrome, deficiency of heart and spleen syndrome, *qi* stagnation and blood stasis syndrome, and *yin* deficiency of heart and liver syndrome. The gender composition (*P*=0.992), age distribution (*F* = 0.700, *P*=0.594), and years of education (*F* = 1.881, *P*=0.118) of the five Chinese medicine syndromes were matched without statistical significance (*P* > 0.05).

### 3.2. MoCA Scores and Cognitive Subitem Scores of Chinese Medicine Syndromes of MCI

Table 2 shows that there were no significant differences in the MoCA scores among different Chinese medicine syndromes (*P* > 0.05). In the kidney deficiency and marrow reduction syndrome, the delayed recall score was 1.74 ± 1.23 and the difference was statistically significant when compared with the deficiency of heart and spleen syndrome or *yin* deficiency of heart and liver syndrome (*P* < 0.05). In the turbid phlegm obstructing orifices syndrome, the delayed recall score was 1.81 ± 1.33 and the difference was statistically significant when compared with the *yin* deficiency of heart and liver syndrome (*P* < 0.05). There were no statistically significant differences in the cognitive subitems scores of the other Chinese medicine syndromes (*P* > 0.05).

The article "Study on the Correlation between Chinese Medicine Syndrome and Cognitive Dysfunction in Mild Cognitive Impairment" was published in 2022. Journal: Evid Based Complement Alternat Med.

### 3.3. Correlation Analysis of Syndrome Scores in Patients with Different Chinese Medicine Syndromes and MoCA Scores or Its Subitem Scores

Table 3 shows that there was a significant negative correlation between the kidney deficiency and marrow reduction syndrome's Chinese medicine syndrome scores and MoCA scores (*R* = −0.570, *P* < 0.01); there was a negative correlation between the turbid phlegm obstructing orifices syndrome's Chinese medicine syndrome scores and MoCA scores (*R* = −0.374, *P* < 0.05). Correlation analysis showed that the kidney deficiency and marrow reduction syndrome was significantly negatively correlated with damage of the delayed recall scores (*R* = −0.558, *P* < 0.01) and it was also negatively correlated with the damage of visual space and executive function scores (*R* = −0.3547, *P* < 0.05). The turbid phlegm obstructing orifices syndrome was significantly negatively correlated with damage of the delayed recall scores (*R* = −0.503, *P* < 0.01).

## 4. Discussion

According to clinical manifestations of MCI, it belongs to the categories of “forgetfulness,” “dullness,” “morbid forgetfulness,” and so on. The disease pathogenesis is essentially empty and out solid, emptying of kidney is the reason, and phlegm and blood stasis are its outer phenomena. In our study, we also found that MCI patients can be manifested as excess syndromes or deficiency syndromes. Generally speaking, deficiency syndromes were more common, which is similar to the results of relevant studies [12–14]. The types of Chinese medicine syndromes from most to least were kidney deficiency and marrow reduction syndrome, turbid phlegm obstructing orifices syndrome, deficiency of heart and spleen syndrome, *qi* stagnation and blood stasis syndrome, and *yin* deficiency of heart and liver syndrome. The kidney deficiency and marrow reduction syndrome and the turbid phlegm obstructing orifices syndrome are the two most common Chinese medicine syndromes, which is consistent with the research results of Liu Xiaoting et al. [15].

Though previous studies have shown that Chinese medicine syndromes may have a certain correlation with cognitive function of MCI patients [16, 17], they still lack systematic evaluation. The MoCA scale is an important neuropsychological tool to screen and evaluate cognition in clinical practice. It is characterized by high sensitivity, specificity, and classification accuracy [11, 18]. In the study, the MoCA scale score was used to evaluate cognitive function of patients with MCI, which improved the credibility of the research results. By analyzing MoCA and subitem scores of different Chinese medicine syndromes, we found that there were no statistical differences in MoCA scores among different Chinese medicine syndromes. There were statistically significant differences in delayed recall among kidney deficiency and marrow reduction syndrome, deficiency of heart and spleen syndrome, and *yin* deficiency of heart and liver syndrome. There were also statistical differences in delayed recall between the turbid phlegm obstructing orifices syndrome and *yin* deficiency of heart and liver syndrome. And, there were no statistically significant differences in other subitem scores between different Chinese medicine syndromes. The wholism concept of TCM holds that the human body is an organic whole, and local lesions are closely related to the functional state of the body. Therefore, we further studied the correlation between Chinese medicine syndrome scores and MoCA scores or subitem scores. Chinese medicine syndrome scores reflect the state of the human body as a whole, it includes not only TCM clinical symptoms, such as a heavy sensation in the head, headache, tinnitus, hypophrenia detail, soreness and weakness of the waist and knees, burnout, night sweats, sleep, defecation and urination, diet, and so on, but also complexion, body, tongue, pulse, and other physical signs. The study indicates that kidney deficiency and marrow reduction syndrome scores or turbid phlegm obstructing orifices syndrome scores have a significant correlation with MoCA scores as well as its subitem scores. For instance, kidney deficiency and marrow reduction syndrome scores were significantly negatively correlated with delayed recall scores, and they were also negatively correlated with visual space and executive function scores. Turbid phlegm obstructing orifices syndrome scores were significantly negatively correlated with delayed recall scores. That is to say that Chinese medicine syndromes of MCI are closely related to cognitive impairment. MCI patients not only had local cognitive domain damage, but also had overall performance of Chinese medicine syndromes. This suggests that we should actively carry out Chinese medicine syndrome differentiation in MCI patients' prevention and treatment, and timely adjust and treat MCI patients' systemic symptoms. It may improve MCI patients' cognitive function.

The article "Study on the Correlation between Chinese Medicine Syndrome and Cognitive Dysfunction in Mild Cognitive Impairment" was published in 2022. Journal: Evid Based Complement Alternat Med.

The results show that there is a significant negative correlation between the kidney deficiency and marrow reduction syndrome and delayed recall, which supports the research results of Liu Yong [19]. It indicates that the worse the deficiency of kidney essence is, the worse the memory is. TCM believes that the kidney is the source of sealing and innate essence, which is the basic substance to stimulate the function of zang-fu organs in the human body. The brain is the house of mentality, and the brain is closely related to the formation of memory function. Whether the function of the brain is normal or not is closely related to the kidney. If the kidney essence is sufficient, the marrow sea will be replenished and nourished and the memory will be strong, otherwise the opposite. It is recorded in *Neijing* that “kidney stores essence, essence gives up Zhi, Zhi injury likes to forget its preface”. *Essentials of Materia Medica* said that “Kidney essence is insufficient, then ambition decline, cannot pass on the heart, so forgetful”. The result is of great significance in guiding MCI syndrome differentiation and treatment, suggesting that we should pay attention to tonifying the kidney in clinical treatment of MCI, especially in delayed recall treatment.

The results show that there is a negative correlation between kidney deficiency and marrow reduction syndrome and visual space/executive function. Executive function is a complex set of abilities that includes willpower, planning, purposeful action, and effective execution. Research has shown that the prefrontal cortex and its connections through the caudate nucleus are the primary sources of the executive function. TCM holds that visual space/executive function is closely related to the eyes, limbs, and brain. The brain is the house of the mentality and the general hub of the executive function. The executive function and visual space are inseparable from the brain's operation and thinking activities. If the brain is full, the visual space and executive function will be agile. If the brain is not full, the function will deteriorate. The results suggest that we need to pay more attention to tonifying the kidney in the clinical treatment of MCI, especially in visual space/executive function treatment, which is consistent with the research results of Fu Hong et al. [20].

The results show that there is a significant negative correlation between the turbid phlegm obstructing orifices syndrome and delayed recall. Various etiologies lead to dysfunction of the spleen in transportation and endogenesis of phlegm. Middle jiao is not transported, the clear air will not rise, and turbidity of *yin* will not fall. Phlegm clouding the clear orifices and upper orifices obstruction lead to forgetfulness. It is recorded in *Danxi's experiential therapy* thatforgetful and short of spirit person have more phlegm. Studies have shown that carriers of ApoE*ε*4 are prone to cognitive impairment, especially memory impairment. ApoE*ε*4 is associated with phlegm syndrome in TCM. Therefore, people with turbidities are more likely to have memory impairment; cognitive functions of patients can be improved obviously by eliminating phlegm and turbidness [21, 22].

The article "Study on the Correlation between Chinese Medicine Syndrome and Cognitive Dysfunction in Mild Cognitive Impairment" was published in 2022. Journal: Evid Based Complement Alternat Med.

The occurrence and development of MCI may show deficiency syndromes or intermingled deficiency and excess syndromes. Clinically, treatment needs to be adjusted according to the actual situation. In consideration of the small samples in this study, we will collect more clinical samples to study the correlation between Chinese medicine syndromes and cognitive dysfunction in MCI.

## Figures and Tables

**Figure 1:** Flow chart of recruitment of participants.

**Table 1:** Baseline characteristics of Chinese medicine syndromes of MCI ($\bar{x}\pm s$).

Chinese medicine syndrome	Kidney deficiency and marrow reduction syndrome	*Yin* deficiency of heart and liver syndrome	Deficiency of heart and spleen syndrome	Turbid phlegm obstructing orifices syndrome	*Qi* stagnation and blood stasis syndrome	F value	*P* value
Case (%)	42 (34.71%)	12 (9.92%)	18 (14.88%)	36 (29.75%)	13 (10.74%)		
Gender (male/female)	20/22	6/6	8/10	19/17	5/8		0.992
Age (years, $\bar{x}\pm s$)	68.38 ± 6.38	66.33 ± 9.43	65.28 ± 7.74	66.53 ± 8.14	67.54 ± 4.37	0.700	0.594
Education (years, $\bar{x}\pm s$)	10.14 ± 3.61	10.33 ± 2.96	10.56 ± 3.07	11.89 ± 3.15	12.00 ± 3.00	1.881	0.118

**Table 2:** Comparison of MoCA and subitem scores among Chinese medicine syndromes ($\bar{x}\pm s$).

Chinese medicine syndrome	MoCA	Visual space and executive function	Naming	Attention	Language	Abstraction	Delayed recall	Orientation
Kidney deficiency and marrow reduction syndrome	22.38 ± 2.12	3.67 ± 0.95	2.64 ± 0.58	5.43 ± 0.70	1.81 ± 0.80	1.24 ± 0.58	1.74 ± 1.23^*∗*^	5.86 ± 0.35
*Yin* deficiency of heart and liver syndrome	22.83 ± 2.76	3.67 ± 1.23	2.50 ± 0.52	5.17 ± 0.72	1.75 ± 1.06	1.08 ± 0.67	2.75 ± 1.49	5.92 ± 0.29
Deficiency of heart and spleen syndrome	23.44 ± 2.04	4.11 ± 1.02	2.72 ± 0.58	5.39 ± 0.85	1.83 ± 0.62	1.28 ± 0.70	2.44 ± 1.20	5.67 ± 0.49
Turbid phlegm obstructing orifices syndrome	22.78 ± 2.04	3.64 ± 0.93	2.61 ± 0.60	5.56 ± 0.61	2.00 ± 0.86	1.36 ± 0.64	1.81 ± 1.33^#^	5.81 ± 0.58
*Qi* stagnation and blood stasis syndrome	23.38 ± 2.40	3.85 ± 1.07	2.69 ± 0.63	5.31 ± 0.63	2.31 ± 0.75	1.38 ± 0.65	1.92 ± 0.86	5.92 ± 0.28

Note: ^*∗*^*P* < 0.05 vs. deficiency of heart and spleen syndrome or *yin* deficiency of heart and liver syndrome, ^#^*P* < 0.05 vs. *yin* deficiency of heart and liver syndrome.

**Table 3:** Correlation analysis of syndrome scores with MoCA and its subitems scores in patients with different chinese medicine syndromes.

Chinese medicine syndrome	MoCA	Visual space and executive function	Naming	Attention	Language	Abstraction	Delayed recall	Orientation
Kidney deficiency and marrow reduction syndrome	−0.570^*∗∗*^	−0.357^*∗*^	−0.188	0.193	−0.150	−0.047	−0.558^*∗∗*^	−0.195
*Yin* deficiency of heart and liver syndrome	0.039	−0.088	−0.312	0.189	0.116	0.163	−0.055	0.330
Deficiency of heart and spleen syndrome	−0.220	0.206	−0.265	−0.190	−0.241	−0.031	−0.085	0.336
Turbid phlegm obstructing orifices syndrome	−0.374^*∗*^	−0.143	0.142	−0.060	−0.155	−0.247	−0.503^*∗∗*^	0.021
*Qi* stagnation and blood stasis syndrome	0.188	0.363	0.410	0.205	−0.172	0.099	−0.299	0.000

Note: Pearson's correlation analysis, ^*∗*^*P* < 0.05, ^*∗∗*^*P* < 0.01.

The article "Study on the Correlation between Chinese Medicine Syndrome and Cognitive Dysfunction in Mild Cognitive Impairment" was published in 2022. Journal: Evid Based Complement Alternat Med.

## Data Availability

Original materials will be made available from the corresponding author upon request and be emailed to applicants requesting original materials within one week.
